# Cancer Detection and Prediction Using Genetic Algorithms

**DOI:** 10.1155/2022/1871841

**Published:** 2022-05-16

**Authors:** Aradhita Bhandari, B. K. Tripathy, Khurram Jawad, Surbhi Bhatia, Mohammad Khalid Imam Rahmani, Arwa Mashat

**Affiliations:** ^1^SITE, VIT, Vellore, Tamil Nadu, India; ^2^College of Computing and Informatics, Saudi Electronic University, Riyadh, Saudi Arabia; ^3^Department of Information Systems, College of Computer Sciences and Information Technology, King Faisal University, Al Hasa, Saudi Arabia; ^4^Faculty of Computing and Information Technology, King Abdulaziz University, Rabigh 21911, Saudi Arabia

## Abstract

Cancer is a wide category of diseases that is caused by the abnormal, uncontrollable growth of cells, and it is the second leading cause of death globally. Screening, early diagnosis, and prediction of recurrence give patients the best possible chance for successful treatment. However, these tests can be expensive and invasive and the results have to be interpreted by experts. Genetic algorithms (GAs) are metaheuristics that belong to the class of evolutionary algorithms. GAs can find the optimal or near-optimal solutions in huge, difficult search spaces and are widely used for search and optimization. This makes them ideal for detecting cancer by creating models to interpret the results of tests, especially noninvasive. In this article, we have comprehensively reviewed the existing literature, analyzed them critically, provided a comparative analysis of the state-of-the-art techniques, and identified the future challenges in the development of such techniques by medical professionals.

## 1. Introduction

*Cancer* is a broad term for a range of diseases that are caused by the uncontrolled proliferation of a body's cells. These cells eventually form a tumor in the body and are likely to invade surrounding tissue or spread throughout the body [1].

*Cancer* is the second leading cause of death globally; lung cancer had the highest mortality rate in 2020, followed by colorectal, liver, stomach, and breast cancers [2]. Major scientific advances over the last thirty years have led to a better understanding of cancer: possible causes, predisposing factors, and possible solutions [3].

As cancer worsens, often exponentially, over time, the early diagnosis of cancer is vital to reducing mortality rates. Unfortunately, screening tests are often invasive and expensive and tracking susceptibility to cancer for each individual is a daunting task [4]. Some of the biggest concerns with cancer screening are cost related, as imaging and blood tests can be expensive and screening tests may not be covered by all insurances, especially in patients who are showing no symptoms [5]. Furthermore, cancer is a family of more than a hundred different diseases that can affect any part of the human body. While some cancer screening tests are widespread, most only focus on specific parts of the body. Finally, cancer is a recurrent disease. Even after complete eradication, it may resurface in individuals, sometimes without any noticeable symptoms. In some types of cancer, especially those related to the breast, recurrence is amongst the greatest factors for high mortality [6].

Machine learning consists of a wide range of algorithms that are programmed to solve problems based on data, often by identifying patterns [7] that are indiscernible to humans. In order to achieve an actionable accuracy, these algorithms are improved either by optimizing the parameters of the machine learning or by reducing irrelevant data by feature selection. Genetic algorithms (GAs) are one class of metaheuristic algorithms that were inspired by biological genetic mechanisms to choose optimal solutions. GAs can be applied either as the base classifier, or as an optimizer for the parameters of base classifiers [8], or as a feature selector on the data.

In order to make cancer-related healthcare optimized and accessible to all, it is important that early detection and noninvasive testing for various types of cancer are widespread and accurate. Since accuracy and efficiency are incredibly important features for any cancer detection process, there is a need for a highly accurate optimization function for parameters and features. Because of this, the metaheuristic GA is a popular field of research for cancer detection and prediction-based algorithms.

This paper presents a systemic review of the applications of genetic algorithms in the detection and prediction of cancer. The various research studies are organized based on the function of the utilized GA. The rest of the research proceeds as follows: Section 2 discusses a background in genetic algorithms in the context of reviewed papers, Section 3 outlines the methodology of the research, Section 4 discusses advances made in cancer prediction and detection using GAs, and Section 5 highlights possible areas for future work before the paper is concluded in Section 6.

## 2. Genetic Algorithms

Genetic algorithms (GAs) are a class of evolutionary algorithms that were developed from a theory of adaptive systems by Holland in 1962 [9]. These algorithms work on the principles of evolution and natural selection as highlighted by Charles Darwin. They search procedures that work on probability and are designed to work on spaces where states can be represented as strings [10]. They are generally used to find high-quality solutions for problems such as selecting optimal parameters or important features.

The execution of GAs is generally perceived in five main functions: generating the initial population, evaluating the “fitness” of the population, selecting the fittest solutions, performing a crossover between the solutions, and possibly mutating the populations. The iteration of the former four functions is considered as one “evolution” [11]. The architecture of a standard genetic algorithm is shown in Figure 1.

To begin with, the GA requires a genetic representation of the search space, traditionally a string or bit array. This must be tailored to the application where the GA is being applied. Similarly, each GA requires a fitness function on which it can evaluate the possible solutions to the problem. The fitness function is meant to determine, based on a single criterion, how close the given solution is to meeting its ideal objective [12]. A desired fitness level for optimal solution is also required; the iteration terminates either when an optimal fitness is achieved or when the specified number of evolutions have been performed.

The *initial population* is a solution set that is randomly generated from the search space. Since GAs were modelled on evolutionary phenomena, the solutions may be referred to as “chromosomes.” The variables in the solutions are likewise “genes.” Usually, the initial population generation is random; however, in cases where an approximate solution is expected to reside in a specific area, the initialization may be forced into that area [13].

Once the population is determined, either by initialization or after the completion of an evolution, the solutions in the population are evaluated based on *fitness functions*. Fitness functions vary according to the problem the GA seeks to solve and are often tailored specifically to one solution space. Two main classes of fitness functions exist, immutable and mutable, where the latter may differentiate the population into niches. In order to make a GA efficient, the fitness function must be computationally efficient and fast and should converge at an appropriate solution. Often, a classifier is run on the chromosome and the fitness is the value of an evaluation criterion such as accuracy or area under ROC curve: in such situations, the GA may be referred to as a wrapper method.

*Selection* is performed to identify the fittest solutions based on the values generated by the fitness functions. There are various methods to conduct this selection. In roulette selection, a random number is chosen and the first encountered individual with a fitness score higher than the random number is chosen in an iterative manner. In stochastic universal sampling, roulette selection is performed in one round by having multiple, equally-spaced search pointers. In tournament selection, the population is randomly split into subsets and the best individual in each is chosen. Other algorithms do not consider any individuals below a certain fitness value for selection. It is important that the chosen selection scheme identifies an ideal number of fittest solutions without compromising the diversity of the data [14].

After the fittest solutions have been identified, they must be used to create a new population for the next stage of evolution. To accomplish this, a genetic operator is applied. In order to maintain diversity and allow for offspring to potentially be better than either parent, crossover followed by mutation is commonly used, although other heuristics also exist.

Several algorithms exist for performing *crossover* on the selected fittest individuals. Parents are randomly chosen, and their genetic information is combined based on the given algorithm. In one-point crossover, the gene sequence at the right of a defined point is swapped between the parents. In two-point crossover, the sequence between the points is swapped, and this can be generalized to k-point crossovers. In uniform crossovers, each bit may be chosen from either of the parents with a given probability [15]. The execution of these crossover functions is shown in Figure 2.

*Mutation* is employed specifically to maintain genetic diversity, specifically to combat premature convergence to a local optimum. In some cases, it may result in an offspring that is mutated and better than either parent. It is often randomized based on a relatively low mutation probability. If the probability is too high, mutations may negate the effects of fitness selection. Various algorithms exist to carry out mutation; however, some are restricted to specific variable types. In bit-string mutation, a single gene in the chromosome will flip at a probability equal to the inverse of its own length. With integer or float type variables, a gene will be replaced with either upper or lower boundary bit randomly. Another mutation for these types is uniform mutation, where the chosen genes are replaced uniformly with a random value that is selected between a specified upper and lower bound for the gene. Gaussian mutations are also popular, where genes are replaced by a Gaussian random distribution variable which is a function of the mean and standard deviation of the gene, given that it lies within specified boundary values. In adaptive mutation [16], the mutation probability of the chromosomes is varied based on their fitness values, so that fitter chromosomes have lower probabilities and less fit chromosomes have higher probabilities of mutation. This decreases the chance of disrupting a high-fitness chromosome while still exploiting the exploratory possibilities of chromosomes if they have lower fitness. Appropriate mutation types must be chosen appropriately for the problem: while adaptive mutation works well for specific problems, static techniques work well for more general problems [17].

### 2.1. General Developments and Improvements in Genetic Algorithms

Katoch et al. [18] elaborated on the various recent developments of genetic algorithms and the possible directions for future research. The paper identified that, while GAs that followed a binary encoding scheme had an incredibly high computational complexity, those that followed real-world encodings widely suffered from premature convergence. Multiobjective GAs (MOGA) rely on multiple fitness functions, often via an optimal Pareto front such that no one fitness function can enhance at the decrement of the other fitness functions. MOGAs allow for more than one outcome to be prioritized, which is necessary in many domains of cancer-based research, such as classification. Finally, GAs have also been combined with other optimization techniques, in order to overcome shortcomings in sampling capability and search capability, replace the genetic operators, or optimize the control parameters.

## 3. Research Methodology

This review was conducted to provide an overview of the applications and effectiveness of GAs in a medical context, specifically related to various types of cancer. This research aimed to answer the following questions:

- What role do genetic algorithms play in the detection and prediction of various cancers?
- How do genetic algorithms compare to other algorithms that may be used for similar purposes?
- In what direction should future research be directed to overcome the shortcomings faced by genetic algorithms in the context of detection and prediction of various cancers?

As the first step of research, prior reviews of GAs in the context of this research were sought out. While no papers were retrieved that fit this criterion perfectly, Ghaheri et al. (2015) discussed the applications of GAs in medicine in general. Their review is divided into various categories from a perspective of healthcare departments; however, various sections in the paper discuss the use of GAs in detection, screening, classification, and outcome prediction for various types of cancers. In order to avoid overlap with this review, only papers published in or after 2015 were considered for the scope of this study. The novelty of this paper lies in the exploration of recent developments in the use of GAs in the field of *Cancer* research since 2015 and the elaboration of the exact specifications of the GAs developed in research.

The search was conducted on papers between 2015 and 2021 based on the two primary keywords, “genetic algorithm” and “cancer,” and the set of secondary keywords (“detection,” “prediction,” “classification,” and “diagnosis”). Preliminary research concluded that most relevant papers included the keywords in their title: if the keywords were present elsewhere in the article, they were often references. Thus, search was conducted based on the presence of the keywords in the titles of the paper. Keyword search was performed in IEEE Xplore, ACM Digital Library, SpringerLink, Elsevier, ScienceDirect, NCBI Database, and arXiv archives. The initial search result revealed 84 papers containing the given keywords in their titles. Certain papers were available from multiple sources and therefore were repeated in this initial search; after removing papers that had an overlap in the title, abstract, and authors, 61 results remained.

The papers were then studied for relevancy to the topic. Papers that failed to develop their application of GAs in the context of cancer research, the specific field of cancer research targeted, and sufficient details about the GAs used were considered irrelevant and therefore excluded. Similar papers were then identified as papers that shared function of genetic algorithm, all utilized algorithms, and broad type of cancer. Of a set of similar papers, the one with the latest publication date was considered for review and the rest were excluded. After this, 35 papers remained. Then, each of the papers was evaluated based on their explanation of the GA: 7 papers that failed to identify procedure used for the 5 major stages of the GA were excluded. The remaining 28 papers were considered for the purpose of this study. These papers are outlined in Table 1.

### 3.1. Methodological Findings

After identification, the papers were categorized based on the main purpose of the research, the function of the utilized GA, and the type of cancer involved. Papers that considered more than 1 type of cancer were classified as “general.” Most papers thus fell in the general category, followed by research primarily focused on breast cancer, as shown in Figure 3. A majority of the considered papers were taken from either Springer, IEEE Xplore, or Elsevier, as shown in Figure 4. Finally, more than a third of the papers utilized GAs for feature selection, as shown in Figure 5.

## 4. Genetic Algorithms in Cancer Research

This section presents a detailed discussion regarding the use of genetic algorithms in cancer detection, prediction, and research on the basis of the selected papers. The papers are organized into subsections based on the function fulfilled by the GAs. In each subsection, the papers are organized by year, from earliest to latest. An overview of the GAs discussed in this section is presented in Table 2, which compares the papers on objective criteria such as the type of cancer discussed, the type of dataset used, the specific configurations of the genetic algorithm, and the purpose fulfilled by the GA.

### 4.1. Genetic Algorithms for Feature Selection in Cancer Research

Of the 28 identified articles, 13 utilized genetic algorithms for feature selection. Feature selection is the process of improving classifier or predictor performance and reducing computational complexity by eliminating variables that do not have a significant effect on the target class. The aim of feature selection is to identify a subset of features that can accurately describe the data in terms of the given problem space. GAs are well researched and documented as powerful feature selectors in various fields. A common implementation of GAs as feature selectors is with binary chromosome bits, where each bit represents whether a specific feature is included or not. The fitness function utilized is often just the predictor performance [49]. When an algorithm is used for feature selection, it is often in cohorts with a classifier such as, but not limited to, Naïve Bayes (NB), *k*-nearest neighbors (k-NN), support vector machines (SVM) [50], decision trees, logistic regression (LR), random forest (RF) [51], or multilayer perceptron networks (MLP).

#### 4.1.1. Genetic Algorithms Used for Feature Selection in Cancer Diagnosis

Li et al. [19] attempted to enhance noninvasive diagnosis of bladder cancer via surface-enhanced Raman spectroscopy (SERS) by using GAs to find significant features for classification. The SERS data are encoded by float point to create chromosomes, and the initial population was created by randomly selecting 6 integers. Linear discriminant analysis (LDA) is used as a classifier for both, the final classification on the selected features and as a part of the fitness function based on accuracy. The top 25% best performing individuals are selected for further rounds, and the bottom 25% are selected for single-point crossover and random single-point mutation. The function terminates after 100 generations. The proposed model was compared with results from an LDA classifier that used principal component analysis (PCA) for feature selection [52]. The model utilizing GAs had an improvement in area under the ROC curve, specificity, and accuracy compared to the PCA model.

Wang et al. [11] aimed to select important features from breast cancer data in order to generate relevant, human-readable rules that can be utilized in cancer diagnosis. They extracted data from digital images in the Wisconsin Breast Cancer Dataset. Initially, 100 samples are randomly drawn from the dataset and one of the 30 conditional attribute values is used to create a self-organizing map neural network (SOM) in an attempt to discretize the continuous data. Then, the initial population is randomly encoded in binary vectors for the GA. The fitness function is a function of the reliability of a decision attribute on a conditional attribute. Selection is via tournament, and the genetic operators are single-point crossover and uniform mutation. Once the GA has run through 100 evolutions, the features are then reduced in terms of their domain using a discernability matrix before they are used to induce rules that can easily be encoded into human-readable language. The generated rules performed better than accuracy obtained by SVM or neurorule methods.

Maleki et al. [29] utilized GAs for feature selection in the context of lung cancer diagnosis. The GA is initialized using a binary random vector where 0 indicates that the feature is not included and 1 indicates that it is. Selection is performed via roulette-wheel, and crossover is single point, while mutation is bit-string. The fitness function is calculated based on an inverse of the misclassification by a k-NN classifier. The dataset used for the model was a lung cancer dataset from the world data website. The proposed method achieved an accuracy of 100% for the multiclass data, which was marginally higher than the accuracy achieved by k-NN classifier without GA using *k* = 6.

#### 4.1.2. Genetic Algorithms Used for Feature Selection in Cancer Classification

Nguyen et al. [20] utilized GAs in wavelet-GA to perform feature selection on data for ovarian, prostate, and premalignant pancreatic cancer, taken from the FDA-NCI Clinical Proteomics Program Databank [53]. Before the GA was applied, Haar wavelet transformation was performed on the mass spectrometer data to obtain wavelet coefficients. The goal was to find 5 suitable wavelets, and therefore, the chromosome size was restricted to 5. The initial population was created by random sampling based on the two-sample *t*-test filter method to ensure that all samples had a significant difference between them. The fitness function utilizes a linear combination of average posterior probability and error rate of the classifier, here, linear discriminant analysis (LDA). Here, the average posterior probability is a product of the posterior probability and the multivariate normal density, and the error rate is the number of incorrectly classified samples divided by the number of total samples. Stochastic uniform selection, scatter crossover based on a random binary vector with a probability of 0.8, and Gaussian mutations were used in the GA. While the features were extracted based on the LDA classifier, NB, k-NN, SVM, MLP, fuzzy ARTMAPs, adaptive network based fuzzy inference system (ANFIS), and AdaBoost were also used to compare the results against the following feature selection algorithms: none, entropy test, Bhattacharyya distance, receiver operating characteristic (ROC) curve, Wilcoxon method [54], principal component analysis (PCA), and sequential search. The performance was evaluated based on area under the ROC curve (AUC), F1-score statistics, and Mutual Information; wavelet-GA outperformed all other considered algorithms significantly, with the best performance with LDA for the ovarian and pancreatic dataset and with MLP for the prostate dataset. Because of these disparate results, further research into possible classifier combinations is required. Moreover, wavelet-GA required much more time for execution and the improvement shown was relatively small on the ovarian and prostate datasets.

Motieghader et al. [21] developed a feature selection model using GAs and Learning Automata (LA), called GALA, which they tested for classification on five microarray datasets having two or more types of leukemia (ALL_AML - Broad Institute, MLL - MLData.org), lymphoma (SRBCT - National Human Genome Research Institute), colon (Computational Intelligence Lab, University of Jinan), or general (Tumors_9, Tumors_11 - GEMS cancer datasets) cancers. GALA is implemented by including a LA controlled reward or penalty stage after mutation. For the GA, the initial population is created randomly with a random number of genes in each chromosome. The fitness was calculated via average performance of an SVM classifier trained of 4/5th of each dataset. To maintain elitism, the top 10% of individuals were always chosen and immediately passed to the next generation. Then, individuals were chosen based on roulette-wheel selection and those individuals were considered for single-point crossover and order-based mutation. The penalty and reward system was applied to data that had undergone at least either crossover or mutation. Here, each chromosome was equivalent to one automaton and its actions were its genes, where each action had an associated memory size that depicted importance. If a gene value was changed, the chromosomes' new fitness value was compared to the old fitness value: if the fitness improved, the associated gene memory size was incremented, else it was decremented. If the gene's memory reached zero, it would be changed to a random value. This resists low fitness mutations and increases the speed of the algorithm. GALA has an exponential time complexity to the power of 5. GALA outperformed all considered models on the Colon and tumor_9 datasets and, however, had similar accuracy to SVM + GA (Li et al. [55]) and binary particle swarm optimization (Mohammad et al. [56]) on the ALL_AML dataset. It was outperformed by Successive Feature Selection with LDA (Sharma et al. [57]) and other algorithms on the SRBCT, MLL, and Tumors_11 datasets [58, 59].

Sayed et al. [22] proposed a nested-GA for high-dimensional microarray data for colon cancer from the following datasets: The Cancer Genome Atlas (https://tcgadata.nci.nih.gov/tcga/), TCGA DNA methylation dataset, and Gene Expression Omnibus (GEO) from NCBI. The nested-GA consists of two layers, an inner and an outer GA. The outer GA (OGA-SVM) utilizes SVM to evaluate its fitness function and is trained to find the best genes from GEO, while the inner GA (IGA-NNW) utilizes neural network based deep learning as a fitness function and is trained on CpG gene sites from TCGA DNA methylation dataset. The algorithm is quite computationally expensive, as a complete run of IGA-NNW is completed in every generation of OGA-SVM; the output of each layer is used to improve the other layer via optimal initializations. That is, apart from the first iteration, the best OGA-SVM chromosomes are used to initialize the IGA-NNW. After fitness calculation, selection is performed via both elitism and roulette-wheel selection. Both crossover and mutation are single point, the latter is random binary. While the nested-GA outperformed both GA-SVM and GA-NNW for all number of selected genes for the DNA methylation set, performance on the other two datasets was not as consistent, with the nested-GA performing better than, equal to, or worse than other algorithms, including k-NN and RF, depending on the number of features selected.

Rani and Devaraj [23] proposed a two-stage hybrid model using GAs called MI-GA on microarray data for colon, ovarian, and lung cancer. The original search space is first reduced using Mutual Information (MI), which is calculated using probability density functions, and conditional or unconditional entropy. A higher MI value is indicative of low uncertainty and is therefore selected by the MI. The MI selects 50 features that are then fed to the GA to randomize the initial population. The GA utilizes a dual and inverse combinator operator with uniform crossover and mutation [47] as well as a back controlled selection operator (BCSO) [46]. Fitness is calculated based on accuracy of an SVM classifier. The MI-GA feature selection outperformed other feature selection methods for an SVM classifier of all 5 kernel functions for the colon dataset. However, while SVM-polynomial had the best performance for lung (10 features) and colon (20 features) cancer datasets; the execution time for the former was substantially higher than other functions. Furthermore, while no function was clearly superior for the ovarian cancer dataset, the quadratic function had a much higher execution time.

Peng et al. [24] proposed a multilayer feature eliminator (MGRFE) that was based on GAs, which was tested on 19 different microarray cancer datasets, including those with class imbalance and multiple classes [60]. MGRFE functions in three stages: search space reduction, precise wrapper search, and multiple k-fold cross-validation. A GA-based recursive feature eliminator (GA-RFE) performs feature selection in every layer. Search space reduction is performed via feature selection first by *t*-test [61], and then, more than 500 features are selected based on maximal information coefficient [62]. During precise wrapper search, the gene set obtained from the previous stage is fed MGRFE, which is multilayer and has a GA-RFE in each layer. The RFE reduces the number of genes considered, while the embedded GA searches for optimal solutions. The GA uses variable-length integer coding for each individual, with a truncation selection method [14] that works on elitism, single-point crossover, and the mutation applied works specifically to eliminate repetitive genes. The fitness function is based on Gaussian Naïve Bayes classifier accuracy and an adjustment coefficient for imbalanced datasets. The model was primarily compared to the McTwo model proposed by Ge et al. [63] and consistently performed slightly better. In some datasets, MGRFE achieved 100% accuracy, which was also achieved by some previous models.

Chuang et al. [25] proposed a model that identified the relationship between High-Order Single-Nucleotide Polymorphism (SNP) Barcodes for breast carcinogenesis pathways. The proposed model, a hybrid Taguchi-genetic algorithm (HTGA), utilizes the statistical methods proposed by Brendell et al. in 1989 [64] after the crossover operation. The chromosomes contained SNP indexes and the genotypes for the selected SNPs, and the initial population was stochastically generated. The fitness function is the difference between the number of cases and controls for the given SNP combination, as a higher difference denotes a higher probability of detecting relevant SNP barcode combinations. Standard tournament style selection is used, followed by a uniform crossover scheme. Before mutation, a level of Taguchi operations is performed: a suitable two-level orthogonal array is chosen for the matric experiment of two random chromosomes, and the function and signal-to-noise-ratio are calculated, following which the effects of different factors are calculated to identify the best chromosome. This is repeated until an expected number of new chromosomes are generated via the Taguchi method. Random single-point mutation is also performed. The termination condition was 1000 iterations. The proposed HTGA algorithm identified SNP barcodes that had a greater difference between case and controls than particle swarm [65], chaotic particle swarm [66], and genetic algorithms [67] on the same dataset.

Saied et al. [26] utilized GAs for data reduction and feature selection to augment Discrete Wavelet Transform (DWT) based k-NN and SVM for classification on microarray datasets of six different types of cancers [68]. First, the microarray data are decomposed using DWT and the decomposed data are used to generate a random initial population. Fitness is calculated based on k-NN classifier accuracy for the given set of features, and selection is based on elitism. Two crossover techniques are used, namely, single-point crossover and multipoint crossover, followed by bit-string mutation. Finally, both k-NN and SVM classifiers were trained on the set of selected features. For both Haar and dp7 DWT, for four datasets, both classifiers achieved 100% accuracy; however, for the colon dataset, SVM achieved only 90% and for the brain dataset, k-NN achieved only 91.67%. The model performed wavelet-based feature selection methods proposed by Li et al. [69] and discrete wavelet-based feature extraction by Bennet et al. [70] on the leukemia and colon cancer datasets.

Bilen et al. [27] proposed a hybrid model using GAs to enhance classification of leukemia based on microarray gene expression data. To improve the efficiency of the model based on the genes selected for learning, the feature selection is done in two stages. In the first stage, statistical wrapper methods, namely, Fisher Correlation, Information Gain [71], and Wilcoxon Rank Sum [54], are used for preliminary feature extraction. Each method identifies a ranking of all the genes that are then tested by Leave-One-Out Cross-Validation (LOOCV) on k-NN for finally selecting the genes from the first stage. In the second stage, the GA then uses the selected genes to encode a random initial population. This population is tested for fitness based on the LOOCV values decided by voting between k-NN, SVM, and NB classifiers separately. Selection is performed via roulette-wheel with multiple-point crossover and uniform mutation. The features selected after both rounds were tested by various classifiers including k-NN, SVM, NB, linear regression, ANN, and RF. Five of the models achieved both accuracy and AUC above 0.95 with relatively low root mean square error. The feature selection method was then compared with previous literature: with just two selected genes, the proposed algorithm achieved 100% accuracy and LOOCV, although most research only outlines one of these two values.

Deng et al. [28] present multiobjective genetic algorithms (MOGA) using XGBoost as a feature selection algorithm for general cancer classification. XGBoost (also class Extreme Gradient Boosting) is an integration of multiple Classification and Regression Trees (CARTS) and is proficient as obtaining the importance of features. MOGA is a GA that can be used to solve the optimization problem of multiple objective functions under certain constraints. The optimization of the various objectives often leads to conflict, which makes it a difficult problem to solve. First, XGBoost was implemented for an initial feature selection. Then, the selected features were encoded into a random binary array. Fitness function was calculated based on predicted accuracy of a k-NN classifier on the chromosomes feature set and selection was via tournament. The model uses uniform crossover and flip-bit mutation. The selected features are then evaluated based on performance of SVM and NB in 10-fold cross-validation using 13 different datasets of different cancers. With both the classifiers, the XGBoost0-MOGA features often had as much, if not slightly more, accuracy than simply using either XGBoost, MOGA, or no feature selector on the data. While the run time of just MOGA was higher than XGBoost-MOGA, both were considerably higher than just XGBoost and other algorithms considered for comparison: Correlation-Based Feature Selection (CFS) [72], Feature Clustering Based Support Vector Machine Recursive Feature Elimination (FCSVM-RFE) [73], and MultiSurf [74]. These three feature selectors were outperformed by the proposed model.

Seddik and Ahmed [30] performed feature reduction for ovarian cancer detection using GAs with PCA to compare. The GA selected features were classified by NN, and the PCA identified features were classified by LDA. The GA model was created using the Global Optimization Toolbox and Bioinformatic Toolbox from MATLAB. The initial population is created by biogacreate, which generated a population matrix where each row is a random sample of features from the given data. The fitness function, biogafit, uses a linear combination of the posteriori probability and error rate to identify classifier performance. Stochastic uniform selection was applied on the populations. The genetic functions were based on gaoptimset, where scattered crossover and Gaussian mutation are default functions. The features selected by the GA function were classified by a neural network, outperforming PCA + LDA which achieved 93%, by achieving an accuracy of 100%.

### 4.2. Genetic Algorithms for Optimizing Parameters for Machine Learning in Cancer Research

Most machine learning models often allow for the variation of important parameters that can alter the results of the learning. These parameters vary according to the model, and each has a different level of effect on the model. A common example of an important parameter is the value of *k* for a k-NN model: if the value is too low or too high, the accuracy of the model will be affected. In some cases, using default or standard parameters may be suitable for the given task; however, in cancer prediction and detection, high accuracy and low false negatives are essential. Parameter optimization may also be referred to as hyperparameter tuning (HPT) where the weights are not involved. Cross-validation scores are often used to estimate the performance of a set of parameters. Some commonly used techniques for HPT other than GAs are grid search, random search, Bayesian optimization, and gradient-based approach. Selected papers that used GAs both for parameter optimization and feature selection were included in this subsection.

#### 4.2.1. Genetic Algorithms for Optimizing Parameters for Machine Learning in Cancer Diagnosis

Alharbi and Tchier [31] used GAs to optimize the parameters of a fuzzy system that was meant to diagnose breast cancer based on images from the Wisconsin Breast Cancer Dataset. The paper utilizes the Pittsburgh approach, where each individual chromosome represents an entire fuzzy system; the population represents various fuzzy systems. The initial population is a randomly generated pool of fuzzy systems. One of the advantages of the Pittsburgh approach is that it allows for multiobjective optimization via variability in the fitness function; here, a linear function of the ratio of correctly diagnosed cases and a negative factor of low confidence is used as the fitness function. Selection is via the stochastic uniform selection method, crossover is single-point, and mutation is flip-bit. In accuracy, the model outperformed [75] but failed to outperform [76]. However, the given approach was able to measure confidence in prediction, which was not covered by previous approaches.

Chauhan and Swami [32] attempted to improve breast cancer prediction via a weighted average GA. Discrete breast cancer data from the Breast Cancer Wisconsin Dataset were utilized for this study. The entire classification process happens in two faces: first, training and accuracy prediction is run on 8 different classification model; then, the GA is used to calculate the weights for the learning model. The different classification techniques tested are SVM, decision tree, Random Forest, linear model, SVMPoly, Neural Network, AdaBoost, and Gaussian Naïve Bayes. Out of these models, SVM, AdaBoost, and RF were chosen for the next phase. Here, the GA is initialized randomly for float encoded vectors to represent weight values. For each classifier, fitness function is created on their own accuracy predicted by cross-validation. Elitism is used as a fitness selection, and both crossover and mutation are random single-point and bit-string, respectively. The GA-based weighted classifiers were compared against the classic models and models using particle swarm optimization (PSO) and differential evolution (DE). The GA-based models outperformed DE-based models in all aspects; however, while the final accuracy of the other three were the same, the GA-based model had the same false negative (FN) rate as PSO and higher FN rate than the classical model. For sensitive problems such as cancer detection, FNs may be unacceptable.

Resmini et al. [36] attempted to improve the efficiency of thermography for breast cancer diagnosis with the use of GAs with SVM. They used thermal images from DMR-IR and the private database of the Federal University of Pernambuco for the study. The entire process is based on two ensembles with GA: the first selects the best models with optimized features and the second selects the set of optimal parameters. First, a bucket of models' approach is created using GAs, where each individual in a population represents a model with their specific parameters. For this stage, uniform crossover is used with string-bit mutation and occasionally uniform mutation to add randomness. Another genetic operator called asexual reproduction is also used: here, one parent produces two offspring where, in the first, each gene is *n*-1 of the parent gene, and in the second, each gene is *n*+1 of the respective parent gene. While selection is normally roulette-wheel based, decimation events may also occur where the same performance has been observed for several generations: here, the elite 10% survive while the rest of the individuals are randomly created. For the next stage, the GA is used as a feature selector with a random binary encoded vector where a 0 bit means the feature is not included. Here, single-point crossover is used with flip-bit mutation, where mutation happens at least once in the strongest and weakest portions of the population. The model was compared to all other models considered in the literature review, and while the proposed methodology worked well, it was outperformed in each of F1-score, accuracy, sensitivity, specificity. and AUC by at least one other model, although the results were not uniform across measures. However, the proposed methodology has the advantage that the application of GA for model selection reduces complexity compared to an exhaustive search, and the model specifically identifies cancer rather than any abnormalities in the breast.

#### 4.2.2. Genetic Algorithms for Optimizing Parameters for Machine Learning in Cancer Classification

Adorada and Wibowo [33] used GAs for both feature selection and parameter optimization of a backpropagation neural network for breast cancer identification (GABPNN). The breast cancer data, in microarray format, were collected, mapped, normalized, and then encoded. The initial population was randomized. The BPANN was cross-validated for each chromosome, and the fitness function was the inverse of the predicted error. Selection was done via elitism and roulette-wheel selection, where chromosomes selected by the former were immediately sent to the next generation. The latter chromosomes then underwent single-point crossover and bit-flip mutation. In each fold of the training process, the GABPNN network is tested to optimize parameters as well. To justify feature selection, the authors compared a version of GABPNN without feature selection to the proposed model, and the proposed model yielded better results. However, the model was not compared to any benchmark models.

Lu et al. [34] proposed a hybrid algorithm combining both AdaBoost and GAs to classify various types of cancers, specifically breast, lung, colon, leukemia, and brain, from their gene expression datasets for UCI repository. The paper introduces the idea of a decision group, which is a group of different classifiers that are randomly selected and run a given number of times to solve the same problem. Here, k-NN, Decision Tress, and NB are used as the decision group and the final result is agreed on by voting. This decision group is used as the base classifier for AdaBoost, and the GA is implemented to optimize the weights of each of the decision groups. The fitness was determined by the function of the accuracy of each of the decision group classifiers. Random single-point crossover and bit-string mutation are used, and elitism is used as a classifier. The AdaBoost-GA algorithm was then compared to various other ensemble methods such as Bagging, RF, Rotation Forest, AdaBoost, AdaBoost-BPNN, AdaBoost-SVM, and AdaBoost-RF. In terms of accuracy, AdaBoost-GA outperformed all other models in each dataset except for lung cancer, in which it came second to AdaBoost-RF, which came second otherwise. Matthews correlation coefficient (MCC) [77] and area under ROC curve (AUC) were also used for comparison: while AdaBoost-GA had the highest AUC value for all datasets, the results with MCC were not as consistent and other classifiers outperformed. The variance was calculated only on colon and brain datasets, and AdaBoost-GA had the lowest variance, indicating the highest stability. However, the time consumed by AdaBoost-GA was at least 10 times more than all algorithms other than AdaBoost-BPNN. Selection is done via index ordering where there is higher probability of selecting more fit individuals. Crossover and mutation probabilities are probabilistic, higher for individuals that have fitness below average.

Taino et al. [37] proposed GAs as a way to improve colorectal cancer identification from histological images. Features were extracted from the images using the RGB scale and using multiple approaches to identify various types of features. The employed GA worked both as a feature selector and a parameter optimizer: each gene consisted of integers that represented a selection method, a classification method, and the number of features considered for the classification. The selection methods were used for feature ranking: T-statistics [78], relief algorithm [79], gain ratio [71], Information Gain [71], and chi-squared [80]. The classifiers considered were k-NN, SVM, MLP, RF, random tree [81], J48 [82], and KStar [83]. The generation of the initial population is completely random inside the constraints of the number of algorithms and features identifying max value of each gene. The fitness function was the average AUC value for the chosen classifier on the chosen parameters run on a given number of iterations. Selection was based only on fitness value: any individuals with a fitness above 0.7 were selected. Crossover performed was two-point crossover, where the points were predefined as before and after the classifier; that is, the classifier was swapped between parents to create offspring. Mutation varied depending on the gene being mutated: for gene 2 and 3, representing the classifier and selection algorithm, flip mutation was used, while creep mutation was applied on the gene representing number of features. Here, creep mutation indicates that the gene value is randomly either incremented or decremented by 1. The models were tested and trained on colorectal and NHL datasets, and for both, the relief selection method was selected for all top results based on AUC. For the former, Random Forest achieved the highest AUC; however, a majority of top 10 results utilized KStar. For the latter, k-NN had the highest AUC and a majority in the top ten AUCs for the NHL dataset. The proposed method was compared to papers in the literature survey that utilized the same dataset: for the colorectal dataset, the proposed model had the second-best accuracy following a polynomial classifier; for the NHL dataset, however, the proposed model failed to outperform other models.

#### 4.2.3. Genetic Algorithms for Optimizing Parameters for Machine Learning in Cancer Prediction

Pan et al. [35] optimized the performance of a backpropagation neural network for oral cancer survival rate prediction via GAs (PGA-BP). PCA and t-SNE are compared for feature selection. The proposed method uses a probabilistic GA that varies mutation and crossover probability based on the fitness value. The number of input layer neurons is consistent with the number of features, and the GA is implemented to optimize the weights of the BPNN. The population is encoded in strings where each individual chromosome represents the weights in the network. The fitness is calculated based on a reciprocal function of the error. The crossover and mutation probabilities are probabilistic, higher for individuals with fitness below average. Crossover is single point, and mutation is calculated based on a function with randomized parameters. The PGA-BP model was compared to normal GA with BPNN and just BPNN, where the proposed model had the best performance.

Hashem and Aboel-Fotouh [38] combined GAs with Random Forest to predict early hepatocellular carcinoma from discrete data collected at Coimbra's Hospital and University Center. 4 classifiers were considered: Naïve Bayes, k-NN, SVM, and RF. The GA was implemented as a specific optimizer for each algorithm: for k-NN, it optimized the number of neighbors and the power parameter; for SVM, it optimized the regularization parameter; and for RF, it worked on the number of trees. The classifiers were then evaluated based on error rate, sensitivity, specificity, and accuracy. The best classifier would then be used to rank the features. The GA had to be defined separately for each of the three classifiers, as the number of parameters to be optimized varied. Fitness was calculated based on the 5 evaluation criteria. The selection criteria were roulette-wheel, crossover method was new generation, and mutation method was uniform. The four models, including the untuned NB, were compared and the RF classifier outperformed others in most of the criteria, except for prevalence which was marginally better for NB, which was not optimized. The GA optimized RF was then used to rank the features of the dataset.

### 4.3. Genetic Algorithms for Rule Reduction in Cancer Research

Rules in data mining and machine intelligence can be thought of as representations of knowledge. These representations are learned, identified, or evolved by models; these rules can then be used to infer or predict knowledge from data. Because of their fixed nature, rule-based models are usually optimized on a single dataset for a single problem. A common example is association rules that show the probability of relationships between data items, often using if-then rules. Because of their iterative nature and ability to find optimal solutions, GAs are efficient at finding a single rule or set of rules that accurately represent the required information for the problem set.

#### 4.3.1. Genetic Algorithms for Rule Reduction in Cancer Gene Discovery

Medina et al. [39] optimized association rules via GAs for colon cancer gene relation discovery (CANGAR). Here, the algorithm is meant to find optimal Quantitative Association Rules (QARs) and the chromosomes are individual representations of rules. Each chromosome had genes that represented antecedents and consequents where two types of consequents were considered: type 1 represented a set of genes in the dataset and type 2 was a final classification rule, representing whether the patient has cancer or not. In order to make QARs rather simple association rules, each gene has a lower and upper limit that can be used to quantify it. Fitness is calculated based on multiple objectives such as support and confidence of the QAR. The selection is performed via elitism. Crossover is uniform, and mutation is randomly chosen, at different probabilities, out of three different policies. In generalization mutation, a gene is removed from either the antecedent or consequent. On the other hand, specialization adds a gene to either antecedent or consequent. Finally, in interval bound mutation, any one gene from either the antecedent or consequent is mutated inside their interval. The paper considered the top 100 of the most frequent genes that appeared more than 20% of times in the CANGAR chosen rules. Hierarchical cluster analysis, biological validation techniques, and information from literature have been used to validate the genes selected by CANGAR. The work does not present a quantification of the results achieved.

#### 4.3.2. Genetic Algorithms for Rule Reduction in Cancer Prediction

Hassoon et al. [40] used a GA to reduce the rule set generated by a Boosted C5.0 classifier for liver cancer prediction in discrete datasets. Encoding of the GA is based on the encoding for rule discovery described by Freitasin [84]. Fitness function is calculated based on a confusion matrix that checks rate of correct and incorrect predictions of both having and not having cancer on the dataset. Selection is uniform, purely based on fitness values. Crossover is single point, and mutation is flip-bit. A comparison function was also used to define a stopping point by noting convergence among generations. The proposed model is compared to Boosted C5.0 without GA, where the proposed model outperformed the previous algorithm on all four considered accounts (specificity, sensitivity, precision, FPR, FDR, F1-score, and accuracy) despite considering only about a fourth of the initially selected rules.

### 4.4. Other Utilizations of Genetic Algorithms in Cancer Research

Paul et al. [41] implemented a hybrid, multiobjective GA to find a Pareto optimal solution for automatic clustering of microarray data for cancer detection. A solution is deemed Pareto optimal if it denies domination from other solutions. This is used to solve for the compacting and overlap-separation method for the fuzzy relational clustering (FRC). The entire approach is called fuzzy relational clustering with nondomination solution genetic algorithm (FRC-NSGA-II). The individuals in the population are binary and represent the variable-length numbers of clusters. The fitness function is a combination of rank for nondominated solutions and crowding distance of the FRC clusters created for the specific chromosome. Selection is tournament based; however, correlation is also calculated so that all selected individuals are not highly correlated. Before the genetic operators are applied, the chromosomes are sorted based on nondomination on two fronts—the first are those that are not dominated by any individuals and the second are dominated by only one individual who is in the former category. Simulated binary crossover and polynomial mutation are utilized in this GA. The proposed model ranked among the top two accuracies for all four cancer microarray datasets considered: leukemia, lymphoma, prostate tumor, and colon.

Chomatek and Duraj et al. [42] utilized GA to detect outliers to improve breast cancer diagnosis. Since the outlier detection is meant to work efficiently with various classifiers, the GA must be multiobjective. The authors tested three previously existing hybrid GAs for this purpose: SPEA2 [85], NSGA-II [86], and PESA-II [87]. The initial population is encoded in a random string vector where each gene contains an identifier of an observation that should be treated as an outlier, and therefore, each chromosome represents a set of outliers. The length of each chromosome can vary, as the number of outliers is not fixed. As the GA is multiobjective, the fitness is a function of three parameters: the average k-nearest distance between the outliers and nonoutliers, the average distance of the centroid from the outlier, and the total number of outliers. Selection is tournament based, with uniform crossover and mutation may happen in one of three ways, each with their own probability, changing the value of one identifier, adding one identifier, and removing one identifier. The Wisconsin breast dataset was used for the experiment in jMetal Java environment. The results were measured based on percentage of correctly identified outliers, accuracy for correct identification, percent of correct observations, and accuracy of incorrectly identified outliers. The obtained results do not vary significantly between the three algorithms; however, the results were not compared to any benchmark algorithms.

Saha et al. [43] implemented GAs to rank human genes, based on likeliness of the specific cancers, from microarray data. The developed approach, called MicroarrayGA, beings from the top P genes selected from Fisher's Discriminant Criteria [88]. Then, the initial population is randomly generated using binary encoding. The fitness value is calculated for each individual by taking the average of the two-tailed *t*-test between the two output types (cancerous or not) for the specific gene. Selection is done based on top 40% elitism, and random selection is used to find genes for uniform crossover and flip-bit mutation. After 100 iterations, the top chromosomes are considered for selecting the top 15 fittest genes. These are classified via an SVM classifier: the proposed algorithm outperformed all other considered algorithms for the prostate and b-cell lymphoma datasets on the five considered measures: accuracy, F-score, G-mean, recall, and precision.

Ronagh and Eshghi [44] proposed a new method to reconstruct microwave tomography images in order to detect breast cancer. In particular, a hybrid combination of GA and particle swarm optimization (PSO) was used to solve the inverse scattering problem in the second stage of reconstruction. The PSO is mostly included to overcome local minima convergence that may sometimes occur with GAs. The utilized GA is binary and the initial population is generated randomly, where each chromosome represents a solution. The fitness is calculated as a function of the scattered field (that is calculated in the first step of image reconstruction), the measures electromagnetic field, and the number of receiver antennas. Selection is performed via elitism, crossover is uniform, and mutation is flip-bit. The proposed algorithm was compared to an algorithm using only GA, and the proposed algorithm achieved a higher accuracy in identifying tissue types and had a shorter runtime.

Kim et al. [45] applied a binary GA with a Joinpoint Regression Model (JRM) in order to study trends in colorectal cancer. The GA worked towards optimizing both the number and the location of the joinpoints. The chromosome consists of a sequence of binary genes where each gene represents a candidate location. The initial population generation is completely random. Selection is done based on linear-rank selection, crossover is single-point, and mutation is uniform. The proposed algorithm portrayed outstanding computational efficiency in detection of a large number of joinpoints.

## 5. Future Work

While genetic algorithms are ideal for searching for an optimal solution for a problem, it has been used to perform feature selection, optimize parameters, and rule reduction. However, there is still much scope for improvement, both in GAs in general and specifically for cancer research. This section elaborates on scope for improvement in order to outline areas for future work.

### 5.1. Fitness Function

One of the most important variables in any GA is the fitness function. The efficiency of the fitness function is essential to a GA: a bad fitness function would prevent convergence, have high computational costs, or simply not solve the problem at hand.

The fitness function must be specifically designed for each GA, and this is often a point of contention for design. It also means that there is often room for improvement in the design of the fitness function. In this survey alone, most considered research utilized some form of cross-validation in the fitness function, especially where features or parameters were being optimized. Obviously, running cross-validation for each chromosome in each generation is an incredibly costly process in terms of computation. This leaves much scope for improvement in current research.

Another commonly used fitness criterion is the statistical *t*-test; however, it is not as robust and applicable to all types of problems. This indicates room for further research into efficient fitness functions for cancer research using genetic algorithms.

### 5.2. Selection Criteria

The selection criteria also play a large role in the computational costs and efficiency of a GA. The most commonly used selection techniques are elitism, roulette-wheel, and tournament. Elitism has an exponential time complexity and increases the risk of convergence to a local optimum: GAs that use elitism require a higher crossover and mutation probability which is often not implemented. While roulette-wheel improves the probability that the selected pool with be divergent, it faces a loss of selection pressure as the pool converges and has an exponential time complexity. Tournament selection is popular as it requires neither scaling nor sorting of population and therefore has linear time complexity; however, it may increase randomness and therefore reduce consistency of output. Elitism has the highest time complexity followed by roulette-wheel. However, these two techniques are most commonly used in cancer research using GAs. Research into the use of other techniques that are not so computationally expensive but still give the desired result is required. Similarly, further research may also be required into the efficiency, use, and combinations of various genetic operators.

### 5.3. Challenges

Adding to the computational costs of GAs is the large search space for the problems where they have been applied. In most studies, for feature selection, the full range of features is selected; for parameter optimization, the entire allowed range is considered; and for rule reduction, the complete set of rules is searched. However, a larger search space often requires more evolutions to reach an optimal solution. If the fixed number of evolutions is set to lower than the required number, the output may be a local optimum or not an optimum at all. Unfortunately, each additional evolution requires that the fitness function be applied to every chromosome, followed by genetic operators on certain selected chromosomes. Preliminarily reducing the search space via a trust-worthy function that has low operation cost may reduce the computational cost of the entire model significantly.

Another concern with GAs is consistency of results. Since GAs are structured to search in such a randomized fashion, there is room for inconsistency between results on similar training on the same dataset. This is especially true because most GAs start from a randomly generated encoded initial population. Consistency of results is important for industrial use, where inconsistency may result in improper diagnosis of a patient's condition. Motieghader et al. [21] and Chuang et al. [25] identified inconsistency of results as one of their major concerns with GA research, particularly in such a sensitive field.

The quality of data available also plays a big role in determining the efficiency of a model in cancer prediction or detection. Since cancer is such a widely research topic, data specific to certain hospitals or areas are generally available. However, these data may be outdated and, in cases where trend analysis is performed, may not be indicative of current trends. Furthermore, quality of lifestyle, healthcare procedures, and access to healthcare vary significantly by country, which need to be considered when a model is being made for industrial use. Another issue is storing and handling such large amounts of data during collection and training, and deciding how much data the model should be trained on and how often retraining may be required. Finally, in many cases, cancer is not identified until it is in a middle or advanced stage, and therefore, most of the data are not conducive to studies on early prediction of cancer.

### 5.4. Open Issues

A large portion of the research in GAs for cancer classification, diagnosis, or prediction has been in the area of feature selection. While many considered papers did achieve an accuracy of 100%, most of them either considered only one specific type of cancer or only performed to 100% accuracy on some of the considered datasets. For efficient industrial use, cancer classifiers or diagnostic tools should be able to identify at least multiple forms of cancer in one organ, if not multiple forms of cancer in one organ. However, this would require a multiobjective fitness function, as well as reformatting of multiple datasets into one larger dataset. Developing a multiobjective fitness function that can achieve 100% accuracy for multiple types of cancer without incurring large overhead computational costs would be a huge breakthrough for the use of GAs in cancer research.

While many classifiers have been used in the studies, many authors have identified that there is further scope for research into efficient classifiers [89]. The classifier used for the fitness function must be cross-validated several times in each generation to calculate the fitness of each individual, which can contribute to a high computational overhead. Furthermore, there are many options for the classifier used for classification, either after feature selection or parameter optimization or both: an ideal classifier [90] would have a 100% accuracy, or at least 0% false negative rate, as well as efficient use of time and memory resources for both training and individual classification. There is also scope for research into novel deep or fuzzy learning techniques that have been successful in other fields [91].

## 6. Conclusion

In conclusion, while GAs have been used to successfully classify, predict, and diagnose various types of cancer to high levels of accuracy, further research is required to truly make them fit for industrial use. To begin with, GAs are computationally expensive, often much more than traditional algorithms: reduction of number of required evolutions or complexity of fitness functions, selection operators, and genetic operators is expected to reduce this gap. Furthermore, current research shows high accuracy in only some types of cancer or requires separately trained models for each type: there is significant scope for more robust models that can classify multiple kinds of cancer and for models in certain cancer types that have not yet been discussed (for example, ocular cancers). Finally, further research may be necessary regarding the classifiers used in conjunction with GAs.

## Figures and Tables

**Figure 1:** Standard workflow of genetic algorithms.

**Figure 2:** Common crossover techniques (single point, double point, and uniform).

**Figure 3:** Types of cancer studied and their relative percentage of occurrences.

**Figure 4:** Publishing sources of the papers.

**Figure 5:** Function of genetic algorithm.

**Table 1:** Type of cancers and respective datasets of the papers considered in this study.

Ref.	Year		Authors	Cancer	Function	Main purpose	Data type
[19]	2015		Li et al.	Bladder	Feature selection	Diagnosis	Surface-enhanced Raman spectroscopy
[20]	2015		Nguyen et al.	General	Feature selection	Classification	Protein chip generated chip
[11]	2016		Wang et al.	Breast	Feature selection	Diagnosis	Microarray
[21]	2017		Motieghader et al.	General	Feature selection	Classification	Microarray
[22]	2019		Sayed et al.	General	Feature selection	Classification	Microarray
[23]		2019	Rani and Devaraj	General	Feature selection	Classification	Microarray
[24]	2019		Peng et al.	General	Feature selection	Classification	Microarray
[25]	2020		Chuang et al.	Breast	Feature selection	Relation identification	SNPs
[26]	2020		Saied et al.	General	Feature selection	Feature selection	Microarray
[27]	2020		Bilen et al.	Leukemia	Feature selection	Classification	Discrete
[28]	2021		Deng et al.	General	Feature selection	Classification	Microarray
[29]	2021		Maleki et al.	Lung	Feature selection	Diagnosis	Digital image
[30]	2021		Farag Seddik and Ahmed	Ovarian	Feature selection	Detection	Discrete
[31]	2017		Alharbi and Tchier	Breast	Optimizing parameters	Diagnosis	Microarray
[32]	2018		Chauhan and Swami	Breast	Optimizing parameters	Prediction	Microarray
[33]	2019		Adorada and Wibowo	Breast	Optimizing parameters	Classification	Microarray
[34]	2019		Lu et al.	General	Optimizing parameters	Classification	Digital image
[35]	2020		Pan et al.	Oral	Optimizing parameters	Outcome prediction	Digital image
[36]	2021		Resmini et al.	Breast	Optimizing parameters	Diagnosis	Discrete
[37]	2021		Taino et al.	Colorectal	Optimizing parameters	Image study	Microarray
[38]	2021		Hashem and Aboel-Fotouh	Liver	Optimizing parameters	Prediction	Discrete
[39]	2016		Medina et al.	Colon	Rule reduction	Gene discovery	Microarray
[40]	2017		Hassoon et al.	Liver	Rule reduction	Prediction	Discrete
[41]	2016		Paul et al.	General	Misc	Clustering	Microarray
[42]	2018		Chomatek and Duraj	Breast	Misc	Diagnosis	Discrete
[43]	2018		Saha et al.	General	Misc	Ranking	Microarray
[44]	2019		Ronagh and Eshghi	Breast	Misc	Detection	Digital image
[45]	2021		Kim et al.	Colorectal	Misc	Trend analysis	Microarray

**Table 2:** Breakdown of the genetic algorithms of the papers considered in this research.

Ref.	Initialization	Fitness function	Selection	Crossover	Mutation	Termination
[19]	Random initialization of 6 integers less than 254	LDA-based leave-one-spectrum-out cross-validation accuracy	Elitism	Single-point	Random single-point	100 generations
[20]	Random sampling on two-sample *t*-test filter method	Linear combination of error rate and average of posterior probability	Stochastic uniform	Scattered crossover based on random binary vector (0.8)	Gaussian	50 generations
[11]	Random binary vector	Function of decision attributes on conditional attributes reliability	Tournament	Single-point	Uniform	100 generations
[21]	Random binary vector	Accuracy during 5-fold cross-validation using SVM	Top 10% and roulette-wheel	Single-point	Order-based	100 generations
[22]	Random or based on OGA-SVM	SVM and neural network accuracy	Elitism and roulette-wheel	Single-point	Single-point binary	Unspecified fixed number
[23]	Randomized from a set of 50 features selected by mutual information	SVM accuracy	Back controlled selection operator (BCSO) [46]	Uniform (0.4–0.85)	Dual and inverse operator [47]	20 generations
[24]	Randomized after search space reduction using *t*-test and maximal information coefficient	Naïve Bayes (NB) classifier accuracy	Truncation [14]	Single-point	Elimination of repetition	Unspecified fixed number
[25]	Stochastic initialization based on encoding schemes	Difference between the number of intersections for cases and controls	Tournament	Uniform	Random single-point	1000 generations
[26]	Random selection after decomposition using discrete wavelet transformation	K-nearest neighbors (k-NN) accuracy	Elitism	Both single-point and k-point	Bit-string	Unspecified fixed number
[27]	Random encoding	Voting between k-NN, SVM, and NB for LOOCV	Roulette-wheel	k-point	Uniform	Unspecified fixed number
[28]	Random binary vector	SVM accuracy	Tournament	Uniform	Bit-flip	Unspecified fixed number
[29]	Random binary vector	Inverse of k-NN misclassification	Roulette-wheel	Single-point	Bit-string	Unspecified fixed number
[30]	Random initialization using biogacreate function	Linear combination of error rate and posteriori probability using biogafit function	Stochastic uniform	Scattered crossover based on random binary vector [0.8]	Gaussian	50 generations
[31]	Random binary vector	Linear function of ratio of correctly diagnosed cases and a negative factor of low confidence	Stochastic uniform	Single-point	Bit-flip	Unspecified fixed number
[32]	Random encoding	SVM, AdaBoost, and NB accuracy	Elitism	Single-point	Bit-string	Unspecified fixed number
[33]	Random binary vector	Inverse of predicted error from backpropagation neural network (BPNN)	Elitism and roulette-wheel	Single-point	Bit-flip	Unspecified fixed number
[34]	Random binary vector	k-NN, NB, and decision trees accuracy	Elitism	Single-point	Bit-flip	Unspecified fixed number
[35]	Random string vector	Reciprocal function of error	Elitism	Single-point	Random single-point	Unspecified fixed number
[36]	Random selection	Area under ROC curve (AUC)	Roulette-wheel with decimation	Uniform or single-point	Bit-string and bit-flip	Unspecified fixed number
[37]	Random vector	Area under ROC curve (AUC)	Truncation (>0.7) [14]	Two-point	Bit-flip and creep [48]	
[38]	Random vector	Function of 5 evaluation criteria such as accuracy and precision	Roulette-wheel	New generation	Uniform	Unspecified fixed number
[39]	Random selection	Support and confidence	Elitism	Uniform	Generalization, specialization, and interval bound	Unspecified fixed number
[40]	Encoding rule discovery	Rate of correct and incorrect predictions	Stochastic uniform	Single-point	Bit-flip	Unspecified fixed number
[41]	Random vector using consequence antecedent	Support and confidence	Elitism	Uniform	Generalization, specialization, and interval bound	Unspecified fixed number
[42]	Random string vector	Combination of number of outliers and distance of outliers from nonoutliers and centroid	Tournament	Uniform	Change value, add new value, and remove random value	Unspecified fixed number
[43]	Random binary vector	Two-tailed *t*-test	Elitism	Uniform	Bit-flip	100 generations
[44]	Random binary vector	Function of scattered field	Elitism	Uniform	Bit-flip	Unspecified fixed number
[45]	Random binary vector	Function based on minimization of join-point similarity	Linear-rank	Single-point	Uniform	Unspecified fixed number

## Data Availability

The data can be made available upon request to the corresponding author.

## References

[1] Cooper G. M., Hausman R. E. (2000). The development and causes of cancer. *The Cell: A Molecular Approach*.

[2] Ferlay J., Colombet M., Soerjomataram I. (2021 August 15). Cancer statistics for the year 2020: an overview. *International Journal of Cancer*.

[3] National Institutes of Health (Us) (2007). Understanding cancer - NIH curriculum supplement series - NCBI bookshelf. NCBI. https://www.ncbi.nlm.nih.gov/books/NBK20362/.

[4] Who (2021). Cancer. World health organization. https://www.who.int/news-room/fact-sheets/detail/cancer.

[5] Wang G. X., Baggett T. P., Pandharipande P. V. (2019 February). Barriers to lung cancer screening engagement from the patient and provider perspective. *Radiology*.

[6] Massafra R., Latorre A., Fanizzi A. (2021 March 11). A clinical decision support system for predicting invasive breast cancer recurrence: preliminary results. *Frontiers in Oncology*.

[7] Tahir M. (2014). *Protein Subcellular Classification Using Machine Learning Approaches*.

[8] Mirza M. T., Khan A., Tahir M., Lee Y. S. (2013). MitProt-Pred: predicting mitochondrial proteins of Plasmodium falciparum parasite using diverse physiochemical properties and ensemble classification. *Computers in Biology and Medicine*.

[9] Holland J. H. (1962 July 1). Outline for a logical theory of adaptive systems. *Journal of the ACM*.

[10] Goldberg D. E., Holland J. H. (1988). Genetic Algorithms and Machine Learning. *Machine Learning*.

[11] Wang Z., Zhang X., Yang W. Rule induction of breast cancer medical diagnose based on combination of rough sets, artificial neutral network and genetic algorithm.

[12] Chakraborty B. Genetic algorithm with fuzzy fitness function for feature selection.

[13] Julstrom B. A. Seeding the population: improved performance in a genetic algorithm for the rectilinear steiner problem.

[14] Blickle T., Thiele L. (1996 December). A comparison of selection schemes used in evolutionary algorithms. *Evolutionary Computation*.

[15] Hasançebi O., Erbatur F. (2000 November 1). Evaluation of crossover techniques in genetic algorithm based optimum structural design. *Computers & Structures*.

[16] Marsili Libelli S., Alba P. (2000 July). Adaptive mutation in genetic algorithms. *Soft Computing*.

[17] Rajakumar B. R. (2013 January 1). Static and adaptive mutation techniques for genetic algorithm: a systematic comparative analysis. *International Journal of Computational Science and Engineering*.

[18] Katoch S., Chauhan S. S., Kumar V. (2020). A review on genetic algorithm: past, present, and future. *Multimedia Tools and Applications*.

[19] Li S., Li L., Zeng Q. (2015 May 7). Characterization and noninvasive diagnosis of bladder cancer with serum surface enhanced Raman spectroscopy and genetic algorithms. *Scientific Reports*.

[20] Nguyen T., Nahavandi S., Creighton D., Khosravi A. (2015 December 21). Mass spectrometry cancer data classification using wavelets and genetic algorithm. *FEBS Letters*.

[21] Motieghader H., Najafi A., Sadeghi B., Masoudi-Nejad A. (2017 January 1). A hybrid gene selection algorithm for microarray cancer classification using genetic algorithm and learning automata. *Informatics in Medicine Unlocked*.

[22] Sayed S., Nassef M., Badr A., Farag I. (2019 May 1). A nested genetic algorithm for feature selection in high-dimensional cancer microarray datasets. *Expert Systems with Applications*.

[23] Jansi Rani M., Devaraj D. (2019 August). Two-stage hybrid gene selection using mutual information and genetic algorithm for cancer data classification. *Journal of Medical Systems*.

[24] Peng C., Wu X., Yuan W., Zhang X., Zhang Y., Li Y. (2021). MGRFE: multilayer recursive feature elimination based on an embedded genetic algorithm for cancer classification. *IEEE/ACM Transactions on Computational Biology and Bioinformatics*.

[25] Chuang L.-Y., Yang C.-S., Yang H.-S., Yang C.-H. (2020 June 17). Identification of high-order single-nucleotide polymorphism barcodes in breast cancer using a hybrid taguchi-genetic algorithm: case-control study. *JMIR Medical Informatics*.

[26] Saeid M. M., Nossair Z. B., Saleh M. A. A microarray cancer classification technique based on discrete wavelet transform for data reduction and genetic algorithm for feature selection.

[27] Bilen M., Işik A. H., Yiğit T. (2020 January 1). A new hybrid and ensemble gene selection approach with an enhanced genetic algorithm for classification of microarray gene expression values on leukemia cancer. *International Journal of Computational Intelligence Systems*.

[28] Deng X., Li M., Deng S., Wang L. (2022 January 13). Hybrid gene selection approach using XGBoost and multi-objective genetic algorithm for cancer classification. *Medical, & Biological Engineering & Computing*.

[29] Maleki N., Zeinali Y., Niaki S. T. A. (2021 February 1). A k-NN method for lung cancer prognosis with the use of a genetic algorithm for feature selection. *Expert Systems with Applications*.

[30] Seddik A. F., Ahmed H. M. (2021). Ovarian cancer detection based on dimensionality reduction techniques and genetic algorithm. https://arxiv.org/abs/2105.01748.

[31] Alharbi A., Tchier F. (2017 April 1). Using a genetic-fuzzy algorithm as a computer aided diagnosis tool on Saudi Arabian breast cancer database. *Mathematical Biosciences*.

[32] Chauhan P., Swami A. Breast cancer prediction using genetic algorithm based ensemble approach.

[33] Adorada A., Wibowo A. Genetic algorithm-based feature selection and optimization of backpropagation neural network parameters for classification of breast cancer using microRNA profiles.

[34] Lu H., Gao H., Ye M., Wang X. (2021). A hybrid ensemble algorithm combining AdaBoost and genetic algorithm for cancer classification with gene expression data. *IEEE/ACM Transactions on Computational Biology and Bioinformatics*.

[35] Pan X., Zhang T., Yang Q., Yang D., Rwigema J.-C., Qi X. S. (2020 August). Survival prediction for oral tongue cancer patients via probabilistic genetic algorithm optimized neural network models. *British Journal of Radiology*.

[36] Resmini R., Silva L., Araujo A. S., Medeiros P., Muchaluat-Saade D., Conci A. (2021 January). Combining genetic algorithms and SVM for breast cancer diagnosis using infrared thermography. *Sensors*.

[37] Taino D. F., Ribeiro M. G., Roberto G. F. (2021 May). Analysis of cancer in histological images: employing an approach based on genetic algorithm. *Pattern Analysis & Applications*.

[38] Hashem E. M., Aboel-fotouh M. R. (2021 May 1). A random forest-genetic algorithm integration approach for hepatocellular carcinoma early prediction. *Annals of the Romanian Society for Cell Biology*.

[39] Medina A. S., Pichardo A. G., García-Heredia J. M., Martínez-Ballesteros M. Discovery of genes implied in cancer by genetic algorithms and association rules.

[40] Hassoon M., Kouhi M. S., Zomorodi-Moghadam M., Abdar M. Rule optimization of boosted c5. 0 classification using genetic algorithm for liver disease prediction.

[41] Paul A. K., Shill P. C., Kundu A. A multi-objective genetic algorithm based fuzzy relational clustering for automatic microarray cancer data clustering.

[42] Chomatek L., Duraj A. Efficient genetic algorithm for breast cancer diagnosis.

[43] Saha S., Das P., Ghosh A., Dey K. N. Ranking of cancer mediating genes: a novel approach using genetic algorithm in DNA microarray gene expression dataset.

[44] Ronagh M., Eshghi M. Hybrid genetic algorithm and particle swarm optimization based microwave tomography for breast cancer detection.

[45] Kim S., Lee S., Choi J. I., Cho H. (2021 February 10). Binary genetic algorithm for optimal joinpoint detection: application to cancer trend analysis. *Statistics in Medicine*.

[46] Kaya M. (2011 June 1). The effects of a new selection operator on the performance of a genetic algorithm. *Applied Mathematics and Computation*.

[47] Shuai X., Zhou X. (2011 January 1). A genetic algorithm based on combination operators. *Procedia Environmental Sciences*.

[48] Corcoran A. L., Sen S. Using real-valued genetic algorithms to evolve rule sets for classification.

[49] Chandrashekar G., Sahin F. (2014 January 1). A survey on feature selection methods. *Computers & Electrical Engineering*.

[50] Tahir M., Khan F., Rahmani M. K. I., Hoang V. T. (2020). Discrimination of Golgi proteins through efficient exploitation of hybrid feature spaces coupled with SMOTE and ensemble of support vector machine. *IEEE Access*.

[51] Tahir M., Khan A., Majid A., Lumini A. (2013). Subcellular localization using fluorescence imagery: utilizing ensemble classification with diverse feature extraction strategies and data balancing. *Applied Soft Computing*.

[52] Barman I., Dingari N. C., Singh G. P., Kumar R., Lang S., Nabi G. (2012 December). Selective sampling using confocal Raman spectroscopy provides enhanced specificity for urinary bladder cancer diagnosis. *Analytical and Bioanalytical Chemistry*.

[53] Center for Cancer Research (2003). Clinical Proteomics Program Databank - Proteomic Patterns. National Cancer Institute. https://home.ccr.cancer.gov/ncifdaproteomics/ppatterns.asp.

[54] Liao C., Li S., Luo Z. Gene selection for cancer classification using Wilcoxon rank sum test and support vector machine.

[55] Li S., Wu X., Hu X. (2008 May). Gene selection using genetic algorithm and support vectors machines. *Soft Computing*.

[56] Mohamad M. S., Omatu S., Deris S., Yoshioka M. (2011 September 12). A modified binary particle swarm optimization for selecting the small subset of informative genes from gene expression data. *IEEE Transactions on Information Technology in Biomedicine*.

[57] Imoto S., Miyano S., Miyano S. (2012). A top-r feature selection algorithm for microarray gene expression data. *IEEE/ACM Transactions on Computational Biology and Bioinformatics*.

[58] Paul D., Su R., Romain M., Sébastien V., Pierre V., Isabelle G. (2017 September 1). Feature selection for outcome prediction in oesophageal cancer using genetic algorithm and random forest classifier. *Computerized Medical Imaging and Graphics*.

[59] Zorkafli M. F., Osman M. K., Isa I. S., Ahmad F., Sulaiman S. N. (2019 January 1). Classification of cervical cancer using hybrid multi-layered perceptron network trained by genetic algorithm. *Procedia Computer Science*.

[60] Peng C., Wu X., Yuan W., Zhang X., Zhang Y., Li Y. (2018). GitHub - pengeace/MGRFE-GaRFE: multilayer recursive feature elimination based on embedded genetic algorithm for cancer classification. https://github.com/Pengeace/MGRFE-GaRFE.

[61] Zhou N., Wang L. (2007 January 1). A modified T-test feature selection method and its application on the HapMap genotype data. *Genomics, Proteomics & Bioinformatics*.

[62] Lin C., Miller T., Dligach D., Plenge R., Karlson E., Savova G. Maximal information coefficient for feature selection for clinical document classification.

[63] Ge R., Zhou M., Luo Y. (2016 December). McTwo: a two-step feature selection algorithm based on maximal information coefficient. *BMC Bioinformatics*.

[64] Disney J., Pridmore W. A., Bendell A. (1989). *Taguchi Methods: Applications in World Industry*.

[65] Wu S.-J., Chuang L.-Y., Lin Y.-D. (2013 July). Particle swarm optimization algorithm for analyzing SNP-SNP interaction of renin-angiotensin system genes against hypertension. *Molecular Biology Reports*.

[66] Chuang L.-Y., Chang H.-W., Lin M.-C., Yang C.-H. (2012 July 1). Chaotic particle swarm optimization for detecting SNP-SNP interactions for CXCL12-related genes in breast cancer prevention. *European Journal of Cancer Prevention*.

[67] Chang W.-C., Fang Y.-Y., Chang H.-W. (2014 December). Identifying association model for single-nucleotide polymorphisms of ORAI1 gene for breast cancer. *Cancer Cell International*.

[68] Bioinformatics Laboratory (2021). University OF ljubljana. https://file.biolab.si/biolab/supp/bi-cancer/projections/.

[69] Li S., Liao C., Kwok J. T. Wavelet-based feature extraction for microarray data classification.

[70] Bennet J., Arul Ganaprakasam C., Arputharaj K. (2014 July). A discrete wavelet based feature extraction and hybrid classification technique for microarray data analysis. *The Scientific World Journal*.

[71] Dai J., Xu Q. (2013 January 1). Attribute selection based on information gain ratio in fuzzy rough set theory with application to tumor classification. *Applied Soft Computing*.

[72] Lu X., Peng X., Deng Y., Feng B., Liu P., Liao B. (2014 February 1). A novel feature selection method based on correlation-based feature selection in cancer recognition. *Journal of Computational and Theoretical Nanoscience*.

[73] Huang X., Zhang L., Wang B., Li F., Zhang Z. (2018 March). Feature clustering based support vector machine recursive feature elimination for gene selection. *Applied Intelligence*.

[74] Urbanowicz R. J., Olson R. S., Schmitt P., Meeker M., Moore J. H. (2018 September 1). Benchmarking relief-based feature selection methods for bioinformatics data mining. *Journal of Biomedical Informatics*.

[75] Setiono R. (1996 February 1). Extracting rules from pruned neural networks for breast cancer diagnosis. *Artificial Intelligence in Medicine*.

[76] Peña-Reyes C. A., Sipper M. (1999 October 1). A fuzzy-genetic approach to breast cancer diagnosis. *Artificial Intelligence in Medicine*.

[77] Boughorbel S., Jarray F., El-Anbari M. (2017 Jun 2). Optimal classifier for imbalanced data using Matthews Correlation Coefficient metric. *PLoS One*.

[78] Meselhy Eltoukhy M., Faye I., Belhaouari Samir B. (2012 January 1). A statistical based feature extraction method for breast cancer diagnosis in digital mammogram using multiresolution representation. *Computers in Biology and Medicine*.

[79] Kira K., Rendell L. A. (1992 January 1). A practical approach to feature selection. *Machine Learning Proceedings 1992*.

[80] Zheng Z., Wu X., Srihari R. (2004 June 1). Feature selection for text categorization on imbalanced data. *ACM Sigkdd Explorations Newsletter*.

[81] Breiman L. (2001 October). Random forests. *Machine Learning*.

[82] Quinlan J. R. (2014 June 28). *C4. 5: Programs for Machine Learning*.

[83] Cleary J. G., Trigg L. E. K: an instance-based learner using an entropic distance measure.

[84] Freitas A. A. (2002 August 21). *Data Mining and Knowledge Discovery with Evolutionary Algorithms*.

[85] Zitzler E., Laumanns M., Thiele L. (2001). SPEA2: improving the strength Pareto evolutionary algorithm. *TIK-report*.

[86] Deb K., Pratap A., Agarwal S., Meyarivan T. (2002 August 7). A fast and elitist multiobjective genetic algorithm: nsga-II. *IEEE Transactions on Evolutionary Computation*.

[87] Corne D. W., Jerram N. R., Knowles J. D., Oates M. J. PESA-II: region-based selection in evolutionary multiobjective optimization.

[88] Iatan I. F. (2010). The Fisher’s linear discriminant. *Combining Soft Computing and Statistical Methods in Data Analysis*.

[89] Reddy G. T., Reddy M. P. K., Lakshmanna K., Rajput D. S., Kaluri R., Srivastava G. (2020). Hybrid genetic algorithm and a fuzzy logic classifier for heart disease diagnosis. *Evolutionary Intelligence*.

[90] Agrawal S., Sarkar S., Alazab M., Maddikunta P. K. R., Gadekallu T. R., Pham Q. V. (2021). Genetic CFL: hyperparameter optimization in clustered federated learning. *Computational Intelligence and Neuroscience*.

[91] Bhalla K., Koundal D., Bhatia S., Khalid Imam Rahmani M., Tahir M. (2022). Fusion of infrared and visible images using fuzzy based siamese convolutional network. *Computers, Materials & Continua*.

